# Risk Factors of Restroke in Patients with Lacunar Cerebral Infarction Using Magnetic Resonance Imaging Image Features under Deep Learning Algorithm

**DOI:** 10.1155/2021/2527595

**Published:** 2021-11-18

**Authors:** Chunli Ma, Hong Li, Kui Zhang, Yuzhu Gao, Lei Yang

**Affiliations:** ^1^Department of Neurology, The Second Affiliated Hospital of Mudanjiang Medical University, Mudanjiang 157010, Heilongjiang, China; ^2^Clinical Skills Training Center, First Clinical Medical College, Mudanjiang Medical University, Mudanjiang 157011, Heilongjiang, China; ^3^Department of Neurology, Mudanjiang Second People's Hospital, Mudanjiang 157013, Heilongjiang, China; ^4^Department of Imaging, Mudanjiang Second People's Hospital, Mudanjiang 157013, Heilongjiang, China

## Abstract

This study was aimed to explore the magnetic resonance imaging (MRI) image features based on the fuzzy local information C-means clustering (FLICM) image segmentation method to analyze the risk factors of restroke in patients with lacunar infarction. In this study, based on the FLICM algorithm, the Canny edge detection algorithm and the Fourier shape descriptor were introduced to optimize the algorithm. The difference of Jaccard coefficient, Dice coefficient, peak signal-to-noise ratio (PSNR), structural similarity index measure (SSIM), running time, and segmentation accuracy of the optimized FLICM algorithm and other algorithms when the brain tissue MRI images were segmented was studied. 36 patients with lacunar infarction were selected as the research objects, and they were divided into a control group (no restroke, 20 cases) and a stroke group (restroke, 16 cases) according to whether the patients had restroke. The differences in MRI imaging characteristics of the two groups of patients were compared, and the risk factors for restroke in lacunar infarction were analyzed by logistic multivariate regression. The results showed that the Jaccard coefficient, Dice coefficient, PSNR value, and SSIM value of the optimized FLICM algorithm for segmenting brain tissue were all higher than those of other algorithms. The shortest running time was 26 s, and the highest accuracy rate was 97.86%. The proportion of patients with a history of hypertension, the proportion of patients with paraventricular white matter lesion (WML) score greater than 2 in the stroke group, the proportion of patients with a deep WML score of 2, and the average age of patients in the stroke group were much higher than those in the control group (*P* < 0.05). Logistic multivariate regression showed that age and history of hypertension were risk factors for restroke after lacunar infarction (*P* < 0.05). It showed that the optimized FLICM algorithm can effectively segment brain MRI images, and the risk factors for restroke in patients with lacunar infarction were age and hypertension history. This study could provide a reference for the diagnosis and prognosis of lacunar infarction.

## 1. Introduction

Lacunar cerebral infarction (LCI) is a common type of ischemic stroke, and LCI patients in China account for more than 25% of cerebral infarction [1]. At present, imaging techniques such as computed tomography (CT) and magnetic resonance imaging (MRI) are often used to diagnose patients with lacunar infarction. When CT is used to diagnose lacunar cerebral infarction, there are low-density changes in the lesion site and the boundary is unclear. At the same time, it is less sensitive to the brain tissue edema caused by lacunar infarction. If the patient undergoes a CT examination less than 24 hours after the onset of the disease, the infarct focus of the brain tissue has not changed significantly at this time, so the positive rate of CT examination is low. MRI is often used in the diagnosis and treatment of intracerebral atherosclerosis due to its noninvasive, simple operation and high resolution [2]. MRI has higher tissue resolution, can clearly display early lesions, and is very sensitive to cytotoxic edema and interstitial edema. The diffusion-weighted imaging (DWI) sequence can show the lesions 3 hours after the onset of lacunar infarction, and low-field MRI scans for lacunar infarctions are significantly better than CT scans [3]. Current research results show that the history of hyperlipidemia, hypertension, diabetes, obesity, and smoking is a risk factor for LCI [4, 5], but the related risk factors for restroke in LCI patients are still unclear.

At present, traditional clustering techniques and deep learning algorithms are often used to segment them. Among them, deep learning shows the advantages of fast calculation, speed, and high accuracy and is widely used in medical image processing [6]. However, in the process of extracting the features of MRI images, the deep learning method requires multiple feature learning training, and it can be applied to the segmentation of the test set image. It ignores the brain structure features [7], so its segmentation accuracy needs to be further improved. Based on the fuzzy local information C-means clustering (FLICM) algorithm in the image segmentation process, not only the domain information of the pixels is considered but also the parameters can be updated through continuous iteration, which can effectively improve the accuracy of image segmentation [8]. However, the FLICM algorithm only uses the characteristics of the image itself in the process of segmenting the middle H-shaped region of the cerebrospinal fluid and does not combine the unique biological structure of the brain, which needs to be further optimized.

In summary, the relevant risk factors for restroke in LCI patients are still unclear, and the FLICM algorithm still has certain limitations in the segmentation of MRI brain tissue. In this study, an MRI image brain tissue segmentation method was established based on the LCM algorithm, and it was applied to the diagnosis of LCI. According to the MRI image features of LCI patients, the relevant risk factors of restroke were evaluated, so as to provide reference for the diagnosis and prognosis of LCI patients.

## 2. Materials and Methods

### 2.1. Brain Tissue Image Segmentation Method Based on the FLICM Algorithm

The FLICM algorithm is a robust image segmentation algorithm based on fuzzy clustering of local spatial information [9]. It can update the parameters through multiple iterations to minimize the objective function. The objective function can be expressed as the following equation:

(1) $$\begin{array}{c} A_{b}=\sum_{i=1}^{n}\overset{m}{\underset{j=1}{\sum }}\left[\mu_{ij}^{b}{\left\|x_{i}-v_{j}\right\|}^{2}+B_{ij}\right]. \end{array}$$

Here, *x*_*i*_ is a vector of *m*, which represents the pixel dataset in the image, and *i*=1,2,…, *n*; *b* refers to the number of categories; *μ*_*ij*_ is the membership function of *x*_*i*_ belonging to the *j*-th category; *v*_*j*_ represents the cluster center of the *j*-th category, and ‖*x*_*i*_ − *v*_*j*_‖ is the Euclidean distance between the two data; and *B*_*ij*_ is the fuzzy factor, which can be calculated as follows:

(2) $$\begin{array}{c} B_{ij}=\sum_{i\in n_{i}}\frac{1}{1+c_{ij}}\left(1-\mu_{ij}\right){\left\|x_{i}-v_{j}\right\|}^{2}. \end{array}$$

In equation (2), *ni* represents a 3 × 3 area centered on pixel *i* and *c*_*ij*_ represents the Euclidean distance between two points.

The calculation methods of the clustering center and the membership function of the FLICM algorithm are given as the following equations:

(3) $$\begin{array}{c} \mu_{ij}=\frac{1}{{\sum_{k=1}^{b}\left[{\left\|x_{i}-v_{j}\right\|}^{2}+B_{ij}/{\left\|x_{i}-v_{k}\right\|}^{2}+B_{ik}\right]}^{1/m-1}}, \end{array}$$

(4) $$\begin{array}{c} v_{j}=\frac{\sum_{i=1}^{n}{\left(\mu_{ij}\right)}^{m}x^{i}}{\sum_{i=1}^{n}{\left(\mu_{ij}\right)}^{m}}. \end{array}$$

The FLICM algorithm can get the initial contour of the level set evolution, but it cannot realize the automatic segmentation of medicine, so the level set method was applied to control its parameters in this study. It was assumed that the target area was *R.* The level set initialization can be expressed as the following equation:

(5) $$\begin{array}{c} \phi \left(x,y\right)=-4\varepsilon \left(0.5-B\right). \end{array}$$

In equation (5), *B*=*R* ≥ *t*_0_ represents the binary image obtained by the target area *R* through the threshold *t*_0_ ∈ [0.1]. The threshold *t*_0_ can be adjusted to make B close to the standard segmentation of the target area. *ε* refers to the adjusted Dirac function. The calculation method to obtain the two evaluation parameters according to the initialization level set *ϕ* could be expressed as follows:

(6) $$\begin{array}{c} \mathrm{Len}\left(\phi \right)=\int \delta \left(\phi \right)dxdy, \end{array}$$

(7) $$\begin{array}{c} \mathrm{Are}\left(\phi \right)=\int H\left(\phi \right)dxdy, \end{array}$$

(8) $$\begin{array}{c} H\left(\phi \right)=\left\{\begin{array}{cc} 1, & \phi \geq 0,\\ 0, & \phi <0. \end{array}\right. \end{array}$$

It was assumed that the ratio of the parameters Len(*ϕ*) and Are(*ϕ*) was *β*; then, *β*=(Len(*ϕ*)/Are(*ϕ*)). The value of *β* was related to the evolution speed of the level set, and each control parameter of the level set can be evaluated by the *β* value.

The brain tissue image segmentation method based on the FLICM algorithm can obtain the initial classification label of each pixel according to the FLICM algorithm, and the segmented image was obtained after the initial classification label processing. The specific process of brain tissue image segmentation based on the FLICM algorithm is shown in Figure 1.

### 2.2. Establishment of a Segmentation Method for the Middle H-Shaped Region in the Cerebrospinal Fluid Based on the FLICM Algorithm

Before the H-shaped region in the cerebrospinal fluid of the MRI image was segmented, the MRI image had to be preprocessed. In addition to the conventional denoising, the preprocessing of brain MRI images also needed to be processed to remove the skull. The Canny edge detection algorithm has a simple processing process, good real time performance, and good anti-interference performance, so it is suitable for edge detection of MRI images [10]. It was supposed that *H*(*x*, *y*) was the impulse response of the boundary [−*ω*, *ω*] filter and *G*(−*x*) was the edge function. The edge response function of the image filtered by *H*(*x*, *y*) can be expressed as the following equation:

(9) $$\begin{array}{c} F_{G}=\int_{-\omega }^{\omega }G\left(-x\right)H\left(x\right)dx. \end{array}$$

The square root of the noise response is expressed as follows:

(10) $$\begin{array}{c} F_{Z}=\sigma \sqrt{\int_{-\omega }^{\omega }H^{2}\left(x\right)dx}. \end{array}$$

In equations (9)∼(10), *σ* represents the uniform difference of Gaussian noise and *F*_*z*_ represents the square root of the noise response.

The edge positioning accuracy *D* is defined as follows:

(11) $$\begin{array}{c} D=\frac{\left|\int_{-\omega }^{\omega }G^{\prime }\left(-x\right)H^{\prime }\left(x\right)dx\right|}{\sigma \sqrt{\int_{-\omega }^{\omega }H^{\prime 2}\left(x\right)dx}}. \end{array}$$

In equation (11), *G*′(−*x*) and *H*′(*x*) are the derivatives of *G*(−*x*) and *H*(*x*, *y*), respectively.

The average distance *S*(*f*) of the zero-crossing point of the impulse response derivative of the detection operator shall satisfy the following condition:

(12) $$\begin{array}{c} S\left(f\right)=\pi \left\{\frac{\int_{-\infty }^{\infty }H^{\prime 2}\left(x\right)dx}{\int_{-\omega }^{\omega }H^{\prime \prime 2}\left(x\right)dx}\right\}. \end{array}$$

In equation (12), *H*^2″^(*x*) is the second derivative of *H*(*x*, *y*).

The smoothing and denoising were performed on the original image *G*(*x*, *y*) to obtain a smooth image *I*(*x*, *y*). It was supposed that the two-dimensional Gaussian function was expressed as follows:

(13) $$\begin{array}{c} G\left(x,y\right)=\frac{1}{2\pi \sigma^{2}}\exp\left(-\frac{x^{2}+y^{2}}{2\sigma^{2}}\right). \end{array}$$

Then, equation (14) could be used to solve the first-order directional derivative of the Gaussian function *G*(*x*, *y*) in direction *n*:

(14) $$\begin{array}{c} G_{n}=\frac{\partial G\left(x,y\right)}{\partial n}=n\nabla G\left(x,y\right). \end{array}$$

Here, *n* is the direction vector and *n*=[cos  *α*/sin  *α*] and ∇G(*x*, *y*) is the gradient vector and $\nabla G\left(x,y\right)=\left[\begin{array}{c} \partial G/\partial x\\ \partial G/\partial y \end{array}\right]$.

The Canny operator was based on two-dimensional convolution ∇*G*(*x*, *y*)*∗f*(*x*, *y*). In order to improve the operation efficiency of the Canny operator, the two-dimensional convolution template of ∇*G*(*x*, *y*) can be decomposed into two one-dimensional filters, namely,

(15) $$\begin{array}{c} \frac{\partial G\left(x,y\right)}{\partial x}=kx*\;\exp\left[\frac{-x^{2}}{2\sigma^{2}}\right]\exp\left[\frac{-y^{2}}{2\sigma^{2}}\right]=H_{1}\left(x\right)H_{2}\left(x\right), \end{array}$$

(16) $$\begin{array}{c} \frac{\partial G\left(x,y\right)}{\partial y}=ky*\;\exp\left[\frac{-y^{2}}{2\sigma^{2}}\right]\exp\left[\frac{-x^{2}}{2\sigma^{2}}\right]=H_{1}\left(y\right)H_{2}\left(y\right). \end{array}$$

Here, $H_{1}\left(x\right)=\sqrt{k}x*\;\exp\left[-x^{2}/2\sigma^{2}\right]$, $H_{2}\left(y\right)=\sqrt{k}*\;\exp\left[-y^{2}/2\sigma^{2}\right]$, $H_{1}\left(y\right)=\sqrt{k}y*\;\exp\left[-y^{2}/2\sigma^{2}\right]$, and $H_{2}\left(x\right)=\sqrt{k}*\;\exp\left[-x^{2}/2\sigma^{2}\right]$. The image *G*(*x*, *y*) is convolved according to equation (16), and then, the following equations could be obtained:

(17) $$\begin{array}{c} E_{x}=\frac{\partial G\left(x,y\right)}{\partial x}*g\left(x,y\right), \end{array}$$

(18) $$\begin{array}{c} E_{y}=\frac{\partial G\left(x,y\right)}{\partial y}*g\left(x,y\right). \end{array}$$

In equations (15)∼(18), *k* is a constant and *σ* is a Gaussian filter parameter. The partial derivatives of the image *g*(*x*, *y*) along the *x* and *y* directions could be written as follows:

(19) $$\begin{array}{c} E_{x}\left(i,j\right)=\frac{\left[I\left(i,j+1\right)-I\left(i,j\right)+I\left(i+1,j+1\right)-I\left(i+1,j\right)\right]}{2}, \end{array}$$

(20) $$\begin{array}{c} E_{y}\left(i,j\right)=\frac{\left[I\left(i,j\right)-I\left(i+1,j\right)+I\left(i,j+1\right)-I\left(i+1,j+1\right)\right]}{2}. \end{array}$$

The gradient magnitude *M*(*i*, *j*) and direction *η*(*i*, *j*) of each pixel (*i*, *j*) in the image can be expressed as the following equations:

(21) $$\begin{array}{c} M\left(i,j\right)=\sqrt{E_{x}^{2}\left(i,j\right)+E_{y}^{2}\left(i,j\right)}. \end{array}$$

(22) $$\begin{array}{c} \eta \left(i,j\right)=\arctan\frac{E_{y}\left(i,j\right)}{E_{x}\left(i,j\right)}. \end{array}$$

The Fourier descriptor is often used to represent the shape features of a single closed curve [11]. The coordinate sequence of the *N* point on the image boundary after moving counterclockwise can be expressed as the following equation:

(23) $$\begin{array}{c} s\left(k\right)=\left[x\left(k\right)y\left(k\right)\right],\;\;k=0,1,\ldots N-1. \end{array}$$

The complex number for each boundary point could be expressed as follows:

(24) $$\begin{array}{c} s\left(k\right)=x\left(k\right)jy\left(k\right),\;k=0,1,\ldots N-1. \end{array}$$

The discrete Fourier transform coefficients can be expressed as the following equation, in which *λ*(*u*) refers to the Fourier descriptor:

(25) $$\begin{array}{c} \lambda \left(u\right)=\frac{1}{N}\overset{N-1}{\underset{k=0}{\sum }}s\left(k\right)e^{-j^{2}/N},\;u=0,1,\ldots N-1. \end{array}$$

After the MRI image was preprocessed, the Fourier shape descriptor and Canny operator were used to identify its H-shaped area to obtain a grayscale histogram. After the threshold range was adjusted to reach the termination condition, the middle H-shaped region segmentation of the cerebrospinal fluid in the MRI image was obtained, and the specific process is shown in Figure 2.

### 2.3. Test Environment and Evaluation of MRI Image Segmentation Performance

The software environment for this experiment was the Windows 10, 64-bit system; the hardware environment was the central processing unit (CPU): Intel (R) Core (TM) i5-8265 U CPU @1.6 GHz, 1.80 GHz; the hard disk was 1040 G; and the memory was 16 G.

The Jaccard coefficient and Dice coefficient were used to evaluate the performance of MRI image segmentation. The Jaccard coefficient represented the degree of coincidence between the segmented image and the standard segmented image, and the value range was [0, 1]. The Dice coefficient was used to evaluate the accuracy of the segmentation algorithm. The calculation methods of the Jaccard coefficient and the Dice coefficient are as follows:

(26) $$\begin{array}{c} \mathrm{Jaccard}=\frac{\left|A_{0}\cap B_{i}\right|}{\left|A_{0}\cup B_{i}\right|}, \end{array}$$

(27) $$\begin{array}{c} \text{Dice }=\;\frac{2\left|A_{0}\cap B_{i}\right|}{\left|A_{0}\right|+\left|B_{i}\right|}. \end{array}$$

The peak signal-to-noise ratio (PSNR) and structural similarity (SSIM) were used to analyze the quality of segmented images. The PSNR is commonly used to evaluate the difference between the image to be tested and the standard image. The calculation method is given as follows:

(28) $$\begin{array}{c} \mathrm{PSNR}\left(A_{0},B_{\text{i}}\right)=10\;\log_{10}\left(\frac{M^{2}}{\mathrm{MSE}\left(A_{0},B_{\text{i}}\right)}\right). \end{array}$$

The SSIM evaluation results were more similar to human senses [12]. The calculation method of SSIM is expressed in the following equation:

(29) $$\begin{array}{c} \mathrm{SSIM}\left(A_{0},B_{\text{i}}\right)=\left(L\left(A_{0},B_{\text{i}}\right)\right)\cdot \left(C\left(A_{0},B_{\text{i}}\right)\right)•\left(S\left(A_{0},B_{\text{i}}\right)\right). \end{array}$$

In equations (28) and (29), *A*_0_ represents the part of the standard segmented image that belongs to category *i*, *B*_*i*_ represents the part of the image segmented by the segmentation algorithm that belongs to category *i*, *M* denotes the peak signal, MSE (*A*_0_, *B*_*i*_) denotes the image mean square error, *L* (*A*_0_, *B*_*i*_) represents the brightness contrast, *C* (*A*_0_, *B*_*i*_) refers to the contrast, and *S* (*A*_0_, *B*_*i*_) refers to the structure contrast.

### 2.4. Research Objects and Their Grouping

36 LCI patients diagnosed in hospitals from February 2019 to June 2020 were selected as the research objects. All patients underwent cranial MRI examination, including 25 males and 11 females. The age range of the patients was 42–86 years, with an average age of 59.45 ± 6.19 years. The inclusion criteria were defined as follows: patients with ischemic stroke with neurological deficit symptoms within one month of onset and patients whose follow-up MRI interval was >2 months. The exclusion criteria were defined as follows: patients with extensive cerebral infarction; patients with a history of malignant tumors; patients with severe liver or renal insufficiency; and patients with a history of mental illness and family history. Patients were divided into a control group (without restroke, 20 cases) and a stroke group (with restroke, 16 cases) according to whether they had restroke. The process had been approved by the ethics committee of the hospital, and all subjects included in the study had signed the informed consent forms.

### 2.5. MRI Examination and Lesion Measurement Method

All patients were examined with a 3.0 TMRI scanner. Diffusion-weighted imaging (DWI) scanning parameters were determined as follows: the time of repetition (TR) was 4100 ms, time of echo (TE) was 102 ms, field of view (FOV) was 230 mm, and layer thickness was 5 mm. The parameters of T2-weighted imaging (T2WI) were determined as follows: TR was 6000 ms, TE was 125 ms, FOV was 240 mm, and layer thickness was 5 mm.

The MRI image scanning and lesion diameter measurement of all patients were completed by a neurologist and an imaging doctor. The diameter of the lesion was measured on the DWI sequence in the MRI image, and the largest diameter was selected through multiple measurements.

### 2.6. Observation Indicators and Standards

The clinical data and imaging characteristics of patients at the time of enrollment were collected. The clinical data included the patient's age, gender, urine protein, and disease history. The MRI features of asymptomatic cerebral infarction (SCI), white matter lesions (WMLs), and perivascular space (PVS) of the patients were collected and measured.

The Fazekas scale [13] was used to evaluate the lateral paraventricular and deep WML scores. The paraventricular WML score can be graded into 4 levels: 0 points (no lesions were seen), 1 point (cap-shaped/pencil linear lesions were visible), 2 points (smooth and ring-shaped lesions were visible), and 3 points (irregular lesions to the deep white matter can be seen). The deep WML score can also be graded into four levels: 0 points (no lesions were seen), 1 point (spotted lesions were visible), 2 points (visible lesions began to merge), and 3 points (large patches of lesions were visible fusion).

### 2.7. Statistical Analysis

The test data were processed using SPSS20.0 statistical software. The mean ± standard deviation ($\bar{x}$ ± *s*) of the measurement data was expressed by the *t*-test, the count data were expressed by the percentage (%), and the *χ*^2^ test was used. *P* < 0.05 indicated that the difference was statistically significant.

## 3. Results

### 3.1. Analysis of the Brain Tissue MRI Image Segmentation Results Based on the FLICM Algorithm

The brain tissue of the original brain MRI image (Figure 3(a)) was segmented by the FLICM algorithm optimized in this study. The segmented brain white matter image (Figure 3(b)), cerebrospinal fluid image (Figure 3(c)), and brain gray matter image (Figure 3(d)) showed that the optimized FLICM algorithm can completely segment different brain tissues from brain MRI images.

### 3.2. Performance of Brain Tissue MRI Image Segmentation Based on the FLICM Algorithm

The optimized FLICM algorithm in this study was compared with the fuzzy C-means algorithm (FCM) and convolutional neural network (CNN) segmentation of brain tissue MRI images of the brain white matter Jaccard coefficients (Figure 4). As the noise level continued to increase, the Jaccard coefficients of different segmentation algorithms showed a downward trend. Under the same noise, the Jaccard coefficient of the optimized FLICM algorithm was remarkably higher than that of the other algorithms.

The optimized FLICM algorithm in this study was compared with the FCM algorithm and CNN algorithm in segmentation of brain tissue MRI images of the brain gray matter Jaccard coefficient (Figure 5). As the noise level continued to increase, the Jaccard coefficients of different algorithms for brain gray matter segmentation all showed a downward trend. Under the same noise, the Jaccard coefficient of the optimized FLICM algorithm was much higher in contrast to that of the other algorithms.

The Dice coefficients in the white matter of brain tissue MRI images with different algorithms were analyzed and compared, and the results are illustrated in Figure 6. As the noise level continued to increase, the Dice coefficients of different algorithms for brain white matter segmentation all showed a downward trend. Under the same noise, the Dice coefficient of the optimized FLICM algorithm was obviously higher than the coefficients of the other algorithms.

The Dice coefficient of gray matter in MRI images of brain tissues with different algorithms was compared, and the results are given in Figure 7. As the noise level continued to increase, the Dice coefficient of gray matter segmentation by different algorithms showed a downward trend. Under the same noise, the Dice coefficient of the optimized FLICM algorithm was obviously higher than that of the other algorithms.

### 3.3. Evaluation of the Segmentation Quality of MRI Images Based on the FLICM Algorithm

The PSNR values of the brain tissue MRI images with different algorithms were compared, and the results are disclosed in Figure 8. As the noise density increased, the PSNR values of the brain tissue MRI image segmentation by different algorithms showed a downward trend. Under the same noise, the PSNR value of the optimized FLICM algorithm was obviously higher than that of the other algorithms.

The SSIM values of brain tissue MRI images with different algorithms were compared, as given in Figure 9. As the noise density increased, the SSIM values of brain tissue MRI image segmentation by different algorithms showed a downward trend. Under the same noise, the SSIM value of the optimized FLICM algorithm was obviously higher in contrast to the values of other algorithms.

### 3.4. Comparison of the Running Time and Segmentation Accuracy of MRI Image Segmentation Based on the FLICM Algorithm

The running time and segmentation accuracy of different algorithms for segmenting the brain tissue MRI images were compared for detailed analysis. As illustrated in Figure 10, the optimized FLICM algorithm showed the shortest running time (26 s) and the highest accuracy (97.86%) for segmenting brain tissue MRI images, which were greatly better than those of the other algorithms, showing statistically obvious differences (*P* < 0.05).

### 3.5. Imaging Characteristics of LCI MRI Images

In the abnormal white matter signal, the T1 sequence showed an equal/low signal (Figure 11(a)) and the T2/flair sequence showed a high signal (Figures 11(b) and 11(c)), with unclear edges and no cavitation in the lesion. A lacunar infarct (shown by the red arrow in the figure) was found on the MRI image, with a diameter of 3 to 15 mm, showing the characteristics of the cerebrospinal fluid signal.

The abnormal perivascular space showed a low signal on the T1-weighted image (T1WI) (Figure 12(a)) and a high signal on the T2-weighted image (T2WI) (Figure 12(b)) on MRI, and the maximum diameter of the lesion was less than 3 mm, which was similar to the signal characteristics of the cerebrospinal fluid (shown by the red arrow in the figure).

WMLs on MRI showed a flair high signal (Figure 13(a)), T1WI low signal (Figure 13(b)), and T2WI high signal (Figure 13(c)), and the lesions were mostly located in the deep white matter of the brain and around the lateral ventricles (shown by the red arrow in the figure).

### 3.6. Risk Factors of LCI Restroke

The gender, age, and disease history of the two groups were compared, and the results are shown in Figure 14. The proportion of patients with a history of hypertension in the stroke group was much higher than that in the control group (*P* < 0.05). There was a great difference in the location of the lesion between the two groups (*P* < 0.05). The proportion of patients with WML scores greater than 2 in the stroke group was higher than that in the control group (*P* < 0.05), and the proportion of patients with deep WML scores of 2 in the stroke group was higher than that in the control group (*P* < 0.05). In addition, the average age of patients in the stroke group was observably higher in contrast to that of the control group (*P* < 0.05).

Logistics was used for multivariate regression analysis (Table 1). Age and history of hypertension were risk factors for LCI restroke (*P* < 0.05). The location of the lesion and the WML score of the lateral ventricle were greater than 2 points, and the deep WMLs score was 2 points, showing no correlation with the occurrence of LCI restroke (*P* > 0.05).

## 4. Discussion

Based on the FLICM algorithm, the level set method was introduced to automatically segment the brain tissue MRI image, and the Canny edge detection algorithm and Fourier shape descriptor were introduced to identify and segment the middle H-shaped area of the cerebrospinal fluid in this study. The results showed that, under different noise levels, the Jaccard coefficient, Dice coefficient, PSNR value, and SSIM value of the optimized FLICM algorithm for brain tissue white matter and gray matter segmentation were higher than those of the FCM and CNN algorithms. It suggested that the optimized FLICM algorithm in this study can effectively improve the segmentation performance and image quality of MRI images. The traditional FCM algorithm does not take into account the spatial information between image pixels, which makes image segmentation less robust, resulting in a severe degradation of noise image segmentation performance [14]. The FLICM algorithm in this study took into account both the image gray information and the spatial position information, so the segmentation performance was greatly improved [15]. The Canny operator has a certain ability to suppress noise [16], which further improves the quality of segmented images. The research results in this study revealed that the shortest running time of the optimized FLICM algorithm to segment brain tissue MRI images was 26 s, and the highest accuracy was 97.86%, which was much better than other algorithms (*P* < 0.05). This is because the introduction of the level set method in the FLICM algorithm reduces the defect of constantly initializing the contour of the curve [17] and increases its segmentation speed and segmentation accuracy. Zavala Bojorquez et al. [18] used wavelet coefficients as the features vector of the image, adopted the principal component analysis (PCA) to reduce the dimensionality of the features vector, and segmented the MRI image after optimizing the parameters of the support vector machine using the genetic algorithm PSO; it was found that the segmentation accuracy was 91.33%. Pereira et al. [19] used the optimized CNN model to segment brain MRI images and found that the segmentation accuracy was 94.2%. The segmentation accuracy of the optimized FLICM algorithm in this study was visibly better than that of these algorithms.

The results of this study indicated that age and history of hypertension are risk factors for LCI restroke (*P* < 0.05). The location of the lesion, lateral paraventricular WML score greater than 2 points, and deep WML score 2 points showed no correlation with LCI restroke (*P* > 0.05). Li et al. [20] pointed out that age and hypertension are risk factors for small vascular disease in patients with LCI, which were similar to the results of this study. WMLs are related to small blood vessel stenosis or occlusion [21], and they are related to factors such as age, genetics, and environmental factors. The WMLs increase the risk of ischemic stroke [22].

## 5. Conclusions

The FLICM algorithm was optimized and applied to the diagnosis and prognosis analysis of LCI patients in this study. The result was that the optimized FLICM algorithm improved the accuracy and speed of MRI image segmentation and age and history of hypertension were risk factors for LCI restroke. However, there were still some shortcomings in this study. There were few cases included in this study, and there may be errors in the analysis of MRI image features. In future work, we will increase the sample size and further analyze the correlation between MRI image features and LCI restroke. In summary, the optimized FLICM algorithm can effectively segment MRI images, and age and history of hypertension were risk factors for LCI restroke. The results of this study could provide a reference for the diagnosis and prognosis of LCI.

## Figures and Tables

**Figure 1:** The brain tissue image segmentation process based on the FLICM algorithm.

**Figure 2:** The specific process for the middle H-shaped region segmentation of the cerebrospinal fluid in the MRI image.

**Figure 3:** The brain tissue MRI image segmentation results based on the FLICM algorithm. (a) The initial MRI image; (b) the segmented brain white matter MRI image; (c) the segmented cerebrospinal fluid MRI image; and (d) the segmented brain gray matter MRI image.

**Figure 4:** Comparison of the Jaccard coefficients of the brain white matter segmentation in MRI images with different algorithms.

**Figure 5:** Comparison of the Jaccard coefficients of the brain gray matter segmentation in MRI images with different algorithms.

**Figure 6:** Comparison of the Dice coefficients of brain gray matter segmentation in MRI images with different algorithms.

**Figure 7:** Comparison of the Dice coefficients of brain gray matter segmentation in MRI images with different algorithms.

**Figure 8:** Comparison of the PSNR value of brain tissue MRI image segmentation with different algorithms.

**Figure 9:** Comparison of the SSIM value of brain tissue MRI image segmentation with different algorithms.

**Figure 10:** Comparison of the running time and segmentation accuracy of different algorithms for segmentation of MRI images. Note: ^∗^suggests that the difference was statistically obvious in contrast to FLICM algorithms (*P* < 0.05).

**Figure 11:** MRI image of asymptomatic cerebral infarction of a male patient aged 45 years. (a), (b), (c) The T1-weighted image, T2-weighted image, and flair manifestation, respectively.

**Figure 12:** The perivascular space MRI image of a male patient aged 58 years. (a), (b) The T1WI and T2WI, respectively.

**Figure 13:** WML MRI image of a patient. (a), (b), (c) The flair manifestation, T1WI, and T2WI, respectively.

**Figure 14:** Comparison of clinical data and MRI image features of the two groups of patients. (a) The comparison of gender and disease history; (b) the comparison of the location of the lesion; (c) and (d) the lateral ventricle WML and deep WML, respectively; and (e) the comparison of age and lesion diameter. Note: ^∗^suggests that the difference was statistically obvious in contrast to the control group (*P* < 0.05).

**Table 1:** Logistic multivariate regression analysis.

Variables	*B* value	OR value	95% CI	*P* value
Age	0.081	1.077	1.026–6.924	0.005
Hypertension	0.952	2.516	0.768–1.043	0.034
Location of the lesion	−0.765	0.412	0.146–1.125	0.062
The WML score of the lateral ventricle ≥2 points	−0.073	0.414	0.024–7.292	0.256
Deep WMLs = 2 points	−0.341	0.656	0.192–2.718	0.608

Note: 95% CI referred to 95% confidential interval.

## Data Availability

The data used to support the findings of this study are available from the corresponding author upon request.

## References

[1] Pei L., Vidyaratne L., Rahman M. M., Iftekharuddin K. M. (2020). Context aware deep learning for brain tumor segmentation, subtype classification, and survival prediction using radiology images. *Scientific Reports*.

[2] Zeineldin R. A., Karar M. E., Coburger J., Wirtz C. R., Burgert O. (2020). DeepSeg: deep neural network framework for automatic brain tumor segmentation using magnetic resonance FLAIR images. *International Journal of Computer Assisted Radiology and Surgery*.

[3] Wu W., Li D., Du J. (2020). An intelligent diagnosis method of brain MRI tumor segmentation using deep convolutional neural network and SVM algorithm. *Computational and Mathematical Methods in Medicine*.

[4] Sato T., Sakai K., Komatsu T. (2020). Risk factors for infarct expansion are different between lacunar and giant lacunar infarction. *Atherosclerosis*.

[5] Zadeh Shirazi A., Fornaciari E., McDonnell M. D. (2020). The application of deep convolutional neural networks to brain cancer images: a survey. *Journal of Personalized Medicine*.

[6] Bousabarah K., Ruge M., Brand J.-S. (2020). Deep convolutional neural networks for automated segmentation of brain metastases trained on clinical data. *Radiation Oncology*.

[7] Kao P.-Y., Shailja S., Jiang J. (2020). Improving patch-based convolutional neural networks for MRI brain tumor segmentation by leveraging location information. *Frontiers in Neuroscience*.

[8] Ren H., Hu T. (2020). A local neighborhood robust fuzzy clustering image segmentation algorithm based on an adaptive feature selection Gaussian mixture model. *Sensors*.

[9] Pham T. X., Siarry P., Oulhadj H. (2019). A multi-objective optimization approach for brain MRI segmentation using fuzzy entropy clustering and region-based active contour methods. *Magnetic Resonance Imaging*.

[10] Li H., Li A., Wang M. (2019). A novel end-to-end brain tumor segmentation method using improved fully convolutional networks. *Computers in Biology and Medicine*.

[11] Wang G., Li W., Ourselin S., Vercauteren T. (2019). Automatic brain tumor segmentation based on cascaded convolutional neural networks with uncertainty estimation. *Frontiers in Computational Neuroscience*.

[12] Shahriari Y., Fidler R., Pelter M. M., Bai Y., Villaroman A., Hu X. (2018). Electrocardiogram signal quality assessment based on structural image similarity metric. *IEEE Transactions on Biomedical Engineering*.

[13] No H.-J., Yi H.-A., Won K. S., Chang H. W., Kim H. W. (2019). Association between white matter lesions and cerebral glucose metabolism in patients with cognitive impairment. *Revista Española de Medicina Nuclear e Imagen Molecular (English Edition)*.

[14] Deng W., Shi Q., Luo K., Yang Y., Ning N. (2019). Brain tumor segmentation based on improved convolutional neural network in combination with non-quantifiable local texture feature. *Journal of Medical Systems*.

[15] Mlynarski P., Delingette H., Criminisi A., Ayache N. (2019). 3D convolutional neural networks for tumor segmentation using long-range 2D context. *Computerized Medical Imaging and Graphics*.

[16] Naceur M. B., Saouli R., Akil M., Kachouri R. (2018). Fully automatic brain tumor segmentation using end-to-end incremental deep neural networks in MRI images. *Computer Methods and Programs in Biomedicine*.

[17] Thaha M. M., Kumar K. P. M., Murugan B. S., Dhanasekeran S., Vijayakarthick P., Selvi A. S. (2019). Brain tumor segmentation using convolutional neural networks in MRI images. *Journal of Medical Systems*.

[18] Zavala Bojorquez J. A., Jodoin P.-M., Bricq S., Walker P. M., Brunotte F., Lalande A. (2019). Automatic classification of tissues on pelvic MRI based on relaxation times and support vector machine. *PLoS One*.

[19] Pereira S., Pinto A., Alves V., Silva C. A. (2016). Brain tumor segmentation using convolutional neural networks in MRI images. *IEEE Transactions on Medical Imaging*.

[20] Li F., Chen Q.-X., Chen Y., Wang G., Peng B., Yao T. (2019). Prevalence and risk factors of microalbuminuria in patients with lacunar infarction. *Postgraduate Medicine*.

[21] Zhou Y.-N., Gao H.-Y., Zhao F.-F. (2020). The study on analysis of risk factors for severity of white matter lesions and its correlation with cerebral microbleeds in the elderly with lacunar infarction. *Medicine (Baltimore)*.

[22] Ryu W. S., Schellingerhout D., Ahn H. S. (2018). Hemispheric asymmetry of white matter hyperintensity in association with lacunar infarction. *Journal of the American Heart Association*.

